The article "Wavelet and Spectral Analysis of Normal and Abnormal Heart Sound for Diagnosing Cardiac Disorders" was published in 2022. Journal: Biomed Res Int.

# Wavelet and Spectral Analysis of Normal and Abnormal Heart Sound for Diagnosing Cardiac Disorders

**DOI:** 10.1155/2022/9092346

**Published:** 2022-07-27

**Authors:** Amzad Hossain, Sharif Uddin, Parinda Rahman, Meratun Junnut Anee, Md Mehedi Hasan Rifat, M. Monir Uddin

**Affiliations:** ^1^Department of Electrical and Computer Engineering, North South University, Dhaka, Bangladesh; ^2^Department of Electrical and Electronic Engineering, Rajshahi University of Engineering & Technology, Rajshahi, Bangladesh; ^3^Department of Mathematics and Physics, North South University, Dhaka, Bangladesh

## Abstract

Body auscultation is a frequent clinical diagnostic procedure used to diagnose heart problems. The key advantage of this clinical method is that it provides a cheap and effective solution that enables medical professionals to interpret heart sounds for the diagnosis of cardiac diseases. Signal processing can quantify the distribution of amplitude and frequency content for diagnostic purposes. In this experiment, the use of signal processing and wavelet analysis in screening cardiac disorders provided enough evidence to distinguish between the heart sounds of a healthy and unhealthy heart. Real-time data was collected using an IoT device, and the noise was reduced using the REES52 sensor. It was found that mean frequency is sufficiently discriminatory to distinguish between a healthy and unhealthy heart, according to features derived from signal amplitude distribution in the time and frequency domain analysis. The results of the present study indicate the adequate discrimination between the characteristics of heart sounds for automatic detection of cardiac problems by signal processing from normal and abnormal heart sounds.

## 1. Introduction

Heart auscultation is a technique used to evaluate the sound wave generated by the heart's mechanical motion [1]. This is a screening technique that is often employed as the main diagnostic tool for heart diseases [2]. Heart disease is a leading reason of death around the globe. In 2016, an anticipated 17.9 million people died prematurely as a result of heart disease, accounting for 31% of all fatalities globally [3]. Heart failures and strokes account for 85% of all cardiovascular disease-related fatalities worldwide [4]. The high death rate is a result of cardiovascular abnormalities that have to be detected early to minimize long-term consequences and heart death prematurely. Most people in their lifetime experience irregular heartbeat or abnormal heartbeat which is known as arrhythmias. Although arrhythmia is harmless in most instances, increased arrhythmias may be caused by other types of heart disease. Heart diseases can be categorized into three different types. Arrhythmia is caused by problems associated with the electrical system [5]. The electrical system regulates a steady heartbeat. Other heart diseases might be caused due to disruption in blood circulation or due to congenital defects [6]. Stroke, heart attack, and cardiomyopathy are examples of such diseases. One of the common electric disorders of the heart is arrhythmias. This begins in the upper chamber's atria. This includes atrial fibrillation (AF or Afib). The upper chambers of the heart beat 300-400 times in a minute. People with AFib experience symptoms like filling up with fluid, shortness of breath, and swelling of hands and legs. They are five times more likely to have a cardiac arrest. Another type of electrical disorder that is similar to AFib is Atrial Flutter (AFL) [7]. This is similar to AFib as it produces a quick pulse in the atria. AFL is triggered by a single circulating electrical wave about 300 times in minutes. The next category of heart disease is circulatory disorders. Myocardial infarction or more commonly known as heart attack is a circulatory disorder. Sudden heart failure can be caused by cardiac diseases which are affected by external constraints. There must be no time delays in the detection of cardiovascular diseases as they are censorious.

The heart sounds can have indicators of the current disorders or warnings about any forthcoming disorder. The indicators can be present randomly throughout the signal if they may be occurring all the time. This type of nonlinearity of heart sounds can be presented using a discrete wavelet transform (DWT). The digital recording of the heart sound that is generated with an electronic stethoscope is called PCG [8]. The technique of listening to the heart sound with a stethoscope is called cardiovascular auscultation which is a simple way of diagnosis. It is used to examine the heart's functioning and performance. The opening and shutting of the atrioventricular, mitral, and tricuspid valves causes unequal blood pressure, high velocity, and slowing of blood circulation.

One of the leading causes of death across the world is cardiac disease [9]. It has to be identified at an early stage in order to have a better cure [10]. However, the lack of medical professionals in developing countries is worsening the problem [11]. While stethoscopes provide easy, efficient, and cheap ways for the physical examination of the human heart, trained medical experts are required. Mortality in rural areas can be prevented through an early and quick automated diagnosis of cardiac diseases. Therefore, a signal analysis-based heart sound analysis can be a significant way for the detection of cardiac diseases without requiring prior medical or professional training [8]. Primary health care centers may benefit from this analysis to detect early signs of cardiac diseases. Some investigations have been carried out toward the automated detection of diseases. This was done by the analysis of auscultation. Particularly in developing countries, the shortage of medical experts causing mortality can be reduced.

The significant contribution of this paper is finding out a way to differentiate between normal and abnormal hearts for automated screening of cardiac disorders. Various domains were studied in order to comprehend and analyze the variations in heart sound. This work is aimed at isolating cardiac and pulmonary sounds. Modulation filters are added to the time-frequency representation of the initial signal reported in the chest. Then, an iterative wavelet decomposition and reconstruction filter algorithm are applied. The lung signals are taken as noise, and all signals are segregated. Then, the signal-to-noise ratio is determined.

The people from rural areas who have no immediate access to any medical care can be benefited from this study. Body auscultation is the basic diagnostic process held by an expert. But in rural areas, there is a scarcity of expert doctors. In that case, this study titled “Wavelet and Spectral Analysis of Normal and Abnormal Heart Sound for Diagnosing Cardiac Disorders” came into action. We can follow the working overview of the proposed system given in Figure 1. By using the proposed system, rural people can get diagnosed whether his/her heart sound is normal or abnormal even without consulting an expert. This proposed system can be used as a primary diagnostic center. If heart sound is found abnormal, he/she will be needed to consult an expert in this field. If sound comes normal, then he will be relieved of stress, as it is very hard and costly for rural people to come every time to a big city and meet a doctor. This system can come in handy in the primary diagnosis of diseases related to the heart.

The paper is organized as follows: Introduction is described in Section 1. Literature Review is explained in Section 2.  Section 3 explains Methodology. Then, in Section 4, Result and Discussion is explained in detail. Finally, Conclusion is described in Section 5. The future work plan has been described in Section 6.

## 2. Literature Review

Previous literature provides us with some insights into the research areas associated with the early detection of heart failures. Automatic heart sound categorization is a potential study area that is now being explored using signal analysis and artificial intelligence techniques. Auscultation of the heartbeat is still inadequate for diagnosing some cardiac diseases [12]. It does not provide the analyzer with both qualitative and quantitative information about the phonocardiogram signals [13, 14]. Singh et al. [10] compared healthy heart sounds and unhealthy heart sounds. The amplitude and frequency element probability distributions were calculated. This was accomplished through the use of signal processing. The results showed that there was adequate differentiation for automated detection of heart diseases using signal processing. Dey et al. [2] used discrete wavelet transform (DWT) on a spectrogram to evaluate and identify the characteristics of the different approximated components. An 82% accuracy was achieved through this method. Kumar et al. [15] used the same method for analyzing the segmented signals, but an algorithm was used to assess only the S3 components of heart sound, and segmentation was performed. The sensitivity was 90.35%, and the specificity was 92.35%. The accuracy of this analysis was shown by Huiying et al. [16] who suggested a 93% correct ratio by using a heart sound segmentation algorithm. It also used DWT to produce envelopes of approximations from the original signal.

The PCG audio recordings of patients were used to expert chronic heart failure (CHF) by Gjoreski et al. [17]. The results which determined CHF phases were compared, and an accuracy of 92% was achieved. The time and the spectral analysis of the signal were used in this research. For continuous observation of the heart, an automated CHF detection device can be calibrated.

Based on wavelet analysis as well as random forest identifier, Qiao et al. [18] introduced a method to classify adolescents' heart sound data. The heart sound segmentation algorithm was used to determine the positions of S1, systole, S2, and diastole, S3. The random forests provided the most accurate classification results. A 3.01% improvement was observed compared to the normal time and frequency analysis of the heart. After that, Cheng and Zhang [19] suggested a self-construct wavelet basis for heart sound denoising. Compared to other traditional wavelets, the experimental results suggested that a heat sound wavelet can filter out the noise while preserving the main characteristics of the signal. A lower mean square error and a higher signal-to-noise ratio were observed.

Some of the key challenges in the classification of heart sound are the segmentation of sounds, creating the distinction between heart and lung sound, and the time shift changes of wavelet transformation. The heart sound segmentation algorithm was used usually, but Das et al. [20] proposed an unsupervised way to detect the positions of S1, and S2 from phonocardiogram (PCG) recordings. The method offered a maximum FI-score of 98% for normal data and 92.5% for abnormal data. Bahreini et al. [21] suggested the use of fractal dimension to identify sounds S1 and S2 using a hidden Markov model. To overcome the challenge, Tsai et al. [22] showed a novel periodicity code deep autoencoder (PC-DAE) approach to create distinction between the heart and lung sounds. However, the extension of this technique requires additional physiological data that is ECG.

Li et al. [23] proposed another system to distinguish between coronary heart disease and valvular disease using wavelet transform. This suggests that there is a necessity to analyze the heart sounds and make clear distinctions for future prediction. The empirical wavelet transformation was divided into 3 modes by Li et al. [24]; a satisfactory rest of Se was found at a percentage of 94.7%. Furthermore, Elamaran et al. [25] analyzed the PCG signals and the execution time of the results was analyzed with Matlab R2016b. Xiao et al. [26] created a computer-aided approach based on deep learning to identify congenital heart defects in children. Using two unique lightweight convolution neural networks, the heart sounds were analyzed. Dwivedi et al. [27] provided a critical analysis and an in-depth review of the ways of automatic identification and classifications of changes in the cardiac cycle. With the help of mobile technology, this may be utilized for illness treatment and monitoring. Data from the wavelet analysis can be used to train SVM classifiers for better diagnosis. However, it is important to ensure that noise is removed to ensure accuracy. The wavelet threshold denoising method was performed on the retained modes by Liu et al. [28]. The findings show that the heart beats' signal-to-noise ratio (SNR) minimizes the root mean square error under various SNR situations.

The heart is one of the most vital organs, and sustaining life is dependent on its ability to beat in a rhythm. Mondal et al. [29] proposed a novel heart sound denoising technique. This introduced a combined framework of wavelet packet transform (WPT) and singular value decomposition (SVD), and the results were found to be satisfactory. Glazova et al. [30] created a monitoring system remotely that monitored asthma patients by analyzing the duration of the tracheal sound. However, the system could not be made fully autonomous. Li et al. [31] applied machine learning algorithms to heart rate variability features from the ECG signal, but the model could be extended to predict SVT events as well. Mishra et al. [32] analyzed the heart sound of the wavelet domains from the screening of cardiac disorders. The detailed approximation coefficient of DWT was analyzed to differentiate between the normal and abnormal heart sounds. Mohammad-Taheri et al. [33] also analyzed a VT and VF detection using the ECG signal's slope. 70% of the dataset was selected for training, and the rest of the dataset was used for testing. Yaseen et al. [9] examine multiple classifications of the heart sound. It suggests an enhanced automated classification system for cardiac diseases. Discrete wavelet transform (DWT) was used for feature extraction from the heart sound signal. For the improvement of accuracy, DWT features were used for categorization and training using DWT. This method showed a 97% accuracy in diagnosing cardiac disorders.

The available algorithms and the experimental data are in a positive direction. Therefore, there is more scope for development in the direction of creating effective models for heart sound-based automated cardiac illness detection. Several methodologies and techniques used by authors prove that there are significant methods that can be employed to find the heart sound across various age groups. This results in early detection and regular monitoring. Some of the techniques included machine learning, deep learning, wavelet analysis, and analysis of PCG signals. However, the limitation that is existent in almost all papers included the challenger of differentiation between heart and lung sound. The differentiation between a healthy heart and an unhealthy heart is done through some parameters. This suggests that there is a gap in the previous literature in examining and differentiating between heart and lung sounds.

## 3. Methodology

### 3.1. Modeling Circuit Device and Data Collecting Process

In this section, the required steps are described to construct the device to collect real-time data. The main component of the circuit stethoscope has been used in this work, and it is essential to collect generated data from the heart. The stethoscope has chest parts in the form of rods that are used (shown in Figure 2) to listen to internal noises, such as heartbeats. An electret condenser microphone is chosen to construct the circuit to amplify the signal measured by the stethoscope. Noise has to be removed from the original signal. In this case, a REES52 sensor is used to filter out the noise from the amplified signal. The vital part of the project is collecting noise-free data from the noisy heart sound. An Arduino Uno is used to process the data. Matlab can read those excel datasets and interpret the sound to signal. The signal was then denoised and ready for further analysis to extract some features of the signal so that we can compare the normal heart sound with abnormal heart sound and come to a decision whether a person is healthy or unhealthy by simply collecting his heart sound.

The total phenomenon has been shown in the block diagram given in Figure 1.

### 3.2. Data Acquisition

After successfully assembling and constructing the circuit, it is programmed to operate and collect data from the heart. The auscultation that is done with an electronic stethoscope is a cost-effective method. The characteristics of the heart sounds on various domains can be explored using this device to identify more differences between healthy hearts and cardiac patients. This paper proved an analysis of heart sounds using various parameter analyses for the automated detection and screening of cardiac disorders. We collected real heart sound data from both medically fit and unfit people. By doing some spectral analysis, we come to a conclusion that there are several differences in feature between healthy and unhealthy sounds.

### 3.3. Data Description

There are accurate live audio recordings of normal and abnormal heart sounds for finding out the relation of healthy and unhealthy heart sounds to make common cardiac diagnoses. Unhealthiness means abnormal heart rhythms (arrhythmia), heart muscle disorders (cardiomyopathy), congenital defects (problems with the formation of the heart and blood vessels that are present from birth), atrial fibrillation, sick sinus syndrome, sinus tachycardia, heart block, heart failure, etc. If any of these problems happens, then the patient's heart sound becomes weak which leads to a decrease in amplitude than a person who is totally free of those diseases. Description of some of the healthy and unhealthy patients from whom we took our heart sound signals is as follows:

(1) Abnormal sounds
  - 24-year-old man, no symptoms, Autism Spectrum Disorder (ASD). Upon examination, the pulses are normal, and the heart's activity is maximum and maybe slightly elevated towards the left sternal border. Observed the left top sternal margin
  - 23-year-old man, asymptomatic, Patent Ductus Arteriosus (PDA). The examination results in noticeably elevated radial and femoral pulses as well as a significantly elevated heart rate. The heart activity was also slightly raised. Observed the left top sternal margin
  - Aortic stenosis, regurgitation, and an elevated heart rate and irregular pulses in a 20-years-old patient. He seems worn out and ill. No prior symptoms, normal historical development in terms of growth
(2) Normal sounds
  - 23-year-old girl, no symptoms, and in good condition, regular medical examination and regular heartbeat and pulse. Used the stethoscope's diaphragm to listen at the left upper sternal border
  - 20-year-old male. No symptoms, standard physical examination, regular bodily habits, normal heartbeat and pulse, and attended to all four regions. Due to microphone noise on the skin, there are a few crackles; listened to the recurrent noises
  - Boy, 19, without symptoms. Routine medical examination of cardiac impulse and pulse that are normal. Listened to the upper left sternal boundary

The comparison of healthy and unhealthy person's heart sound is shown in Result and Discussion. There are clear findings that a healthy person's heart sound is always greater in amplitude, variance, and energy than that of an unhealthy person. It is understandable that if amplitude is greater, then a healthy man's mean value will also be greater. And these mean, variance, and energy are differentiating criteria between healthy and unhealthy people.

### 3.4. Successive Denoising Process

Figures 3(a)–3(e) show the detailed denoising process step by step. The REES52 sensor was used to filter out the noise from the amplified signal of the stethoscope. Then, this signal is taken as input to Matlab. Wavelet decomposition offers a higher signal analysis. Wavelet decomposition level was chosen as per the criteria of a noise-free signal. After wavelet transform, the majority of the noise data and very little signal data are found in the high-frequency subbands. Here, the various subbands are subjected to gentle thresholding. Lastly, wavelet reconstruction of the signal was attained by wave-rec.

Soft thresholding is used here so that our information does not get cut out unexpectedly. Only the noise signal will be cut out from the original heart sound. Different level of thresholding explains throughout the steps of noise removal from the signal. It is the second phase of noise removal as the first phase of noise removal was done by REES52.

### 3.5. Parameters for Relative Analysis of Healthy and Unhealthy Heart Sound

1. Signal: two different signals are found from healthy and unhealthy subjects. They differ in amplitude and frequency. Healthy signals show much higher amplitude than unhealthy heart signals
2. Spectrogram: healthy heart sound shows higher magnitude with constant variation in magnitude as time progresses. On the other hand, unhealthy subjects are more consistent with magnitude and small in value
3. Normal distribution: according to the normal distribution, data that are close to the mean happen more commonly than data that are far from the mean. Symmetric with respect to the mean
4. Detailed coefficient (cD): denoising of collected heart signals is done so that analysis of heart sound is accurate and efficient. Symlet wavelet levels 1 to 4 are being used here. Healthy and unhealthy heart sounds showed a difference in character and were easy to differentiate between them
5. Approximation coefficient (cA): noise-free signal wavelet levels are much more accurate than noisy signal symlet levels. Healthy and unhealthy signals present different characteristics even after being denoised. So, we can count the approximation coefficient of heart sound also as a differentiating factor between healthy and unhealthy people

So, we came to the conclusion that healthy and unhealthy sound signals show different characteristics and there are enough parameters to differentiate between them. It encourages us to analyze further to extract many more differences between them. We found some factors to differentiate between them as follows:

#### 3.5.1. Mean Value

The threshold level is found about 0.07-0.09 to differentiate between them. If a signal poses a higher mean value of 0.09, then it is healthy; if it is less than 0.07, the person is unhealthy.

#### 3.5.2. Variance

If the variance of a heart sound is above 0.015, it is healthy. On the other hand, if the variance value is less than 0.01, it will be tagged as unhealthy.

#### 3.5.3. Energy of DWT

The energy of discrete wavelet transform coefficient is derived by the simple equation of energy, energy = ∑_*i*=1_^*n*^(*x*)^2^/*n*. Here, *n* = no.of heart sample. *x* = signal amplitude. We found the threshold value of 2*e* − 08 to 0.5*e* − 05 for differentiating between them. Unhealthy samples' energy is much lower than the energy of healthy samples. So, this energy is being counted as a differentiating factor between healthy and unhealthy samples of the heart sound. If a signal has more than 0.5*e* − 05 value, then the person is healthy, and if it is less than 2*e* − 08, the person is unhealthy.

## 4. Result and Discussion

The wavelet domain was studied to understand and interpret the variations in heart sound. The characteristics of the heart vibrations are analyzed using the signal and discrete wavelet transform analysis. In this section, real-time data collected by the proposed device will be presented with appropriate figures. Real data was found through a stethoscope with some electronic devices. Body auscultation is one of the most important clinical testing methods for the examination of cardiac disorders. This medicinal approach is inexpensive and efficient and allows trained physicians to recognize and analyze the sound of the heart for diagnosis. But in the rural areas of Bangladesh, there is a scarcity of medical experts who can give a proper interpretation of heart sounds. To overcome this obstacle, the stethoscope heart sound was converted into an electrical signal via a condenser microphone and then PLX-DAQ tools. PLX-DAQ converted serial monitor data of Arduino into Excel data file. Matlab interpreted the sound to signal. The denoised signal was then plotted, and a comparison of the normal heart sound with abnormal heart sound was conducted. Using the visual comparison, the decision on whether a person is healthy or unhealthy was taken by simply collecting his heart sound.

### 4.1. Signal Analysis

Figure 4(a) is an electrical signal converted from sound recorded from a healthy person. Heart sounds were interpreted as electrical signals in the time domain. This representation of sound can extract various features of sound. It can be seen from the heart's lub dub in these figures. Figure 4(b) represents the electrical signal recorded from an unhealthy person in the time domain. The difference between healthy and unhealthy heart sounds in amplitude was seen. A clear visualization can be seen of the differences between healthy and unhealthy subjects. Figure 4(c) shows such a comparison, and the variation in amplitude and frequency of these signals can be seen. A healthy person shows much higher amplitude than an unhealthy person's signal. Unhealthy and healthy sound visual signals might look so close, but there will always be differences in their magnitude as to mean value.

### 4.2. Spectrogram Analysis

Quadratic time-frequency analysis methods produce spectrograms, which are 2D matrices. Figures 5 and 6 show such spectral signals from healthy and unhealthy subjects.  Figure 6 shows the intensity of the frequency content of the signal as time progresses. We can see that Figure 5 shows a higher magnitude with constant variation in magnitude as time progresses.  Figure 6 is more consistent with magnitude and small in value. We have seen lower magnitude values all around the spectrogram. A clear indication of differences between these figures is noticeable. Singh et al. [10] found a similar result.

### 4.3. Normal Distribution

The probability distribution of heart sounds recorded from a healthy and unhealthy subject with normal distribution predicts the probability of subjects being healthy or unhealthy. Figures 7 and 8 show the probability distribution of healthy and unhealthy subjects. The normal distribution is a continuous probability distribution that has a bell curve probability density function. It is clearly seen that the probability distribution of healthy sample (Figure 7) has a higher density where the unhealthy signal (Figure 8) has a lower density which indicates clear discrimination among healthy and unhealthy samples. That means, it is evident that probability distribution analysis is an important parameter for diagnosing cardiac diseases easily.

### 4.4. Detailed Coefficient (cD): Wavelet Family Sym4 Is Used Here

The detailed coefficient for healthy and unhealthy subjects: Figures 9 and 10 show detailed coefficients taken from a healthy and unhealthy person's cardiopulmonary system, respectively. The gathered cardiac signals are denoised so that future analysis of heart sounds can be precise and efficient. To improve responsiveness, symlet wavelet families are employed. Numerous symlet levels have been tested ranging from 1 to 4 and discovered that level 4 produced the best results. These graphs highlight the differences between these two signals. As a result, we may use the detailed coefficient of heart sound to distinguish between healthy and unwell persons. Figures 11–14 depict four distinct levels of the symlet wavelet family employing precise coefficients for the discrete wavelet transform. As the level goes from 1 to 4, the signal's accuracy improves, and undesirable noise is efficiently eliminated. The variations in levels have been noticed before and after denoising. Noise-free signal wavelet levels are far preferable to noisy signal symlet levels. Before and after denoising, good and unhealthy signals exhibit distinct properties.

### 4.5. Approximation Coefficient (cA)

Wavelet family Sym4 is used here. Approximation coefficient of a healthy and unhealthy subject: Figures 15 and 16 show the denoised approximation coefficient using Sym4 level 4 of a healthy subject and the denoised approximation coefficient using Sym4 level 4 of an unhealthy subject, respectively. Here, approximation coefficients for the heart sound signals of a healthy and unhealthy person are retrieved. To ensure the analysis of heart sound is precise and effective, the gathered cardiac signals are denoised. Here, symlet wavelet families have been used for improved response. Various symlet levels have been used from level 1 to level 4, and level 4 produced the best results. These figures demonstrate the distinct disparities between these two signals. As a result, the heart sound approximation coefficient may be used to distinguish between healthy as well as unhealthy individuals. Figures 17–20 display four distinct levels of the symlet wavelet family utilizing the discrete wavelet transform's exact coefficients. From level 1 to level 4, the accuracy of the signal improves, and unnecessary noise is effectively eliminated.

Additionally, the variations in levels before and after denoising are visible. Compared to noisy signal symlet levels, noise-free signal wavelet levels are substantially more accurate.

After being denoised, good and sick signals exhibit different features. The heart sounds are converted from the spatial domain here to the wavelet domain in the suggested wavelet analysis to obtain more noticeable characteristics. The wavelet initial level decomposition of the heart sound was performed using the symlet filter. The heart sound signal is separated into approximate and precise coefficients using a wavelet. A single number has been computed as a characteristic feature because the range of the amplitude dispersion of the signal in the time and wavelet domain exhibits discriminating behavior for screening of heart diseases. The value of energy of wavelet coefficients can be able to distinguish between healthy and unhealthy heart sounds because the range of amplitude is varied.

Therefore, the mean, variance, and energy value of the heart sound signal's wavelet coefficients are taken into account when determining a person's level of health.

### 4.6. Mean Value Comparison and Threshold Determination

Figure 21 shows the mean value comparison between healthy and unhealthy subjects. Recorded sound signals from healthy and unhealthy people show a wide variety of mean values. Although we have successfully found a threshold value range as an isolation line between healthy and unhealthy subjects, the mean value is not the same for all healthy values. Mean value variation is found due to different gender, age, body structure, etc. So, when we can collect the heart sound data through the data acquisition technique described above, then by finding out the mean value of the recorded sound signal, we can tell whether the person is healthy or unhealthy. The threshold level is found about 0.07-0.09 to differentiate between them.

### 4.7. Variance Comparison and Threshold Determination

Figure 22 shows the variance comparison between healthy and unhealthy heart sounds. According to this present analysis, if the variance of a heart sound is above 0.015, it is unhealthy. On the other hand, if the variance value is less than 0.01, it will be tagged as healthy. A similar result has been observed in [10].

### 4.8. Energy of DWT Coefficient

Figures 23 and 24 show the energy of DWT coefficient of healthy and unhealthy subjects and detailed view of energy of DWT coefficient of unhealthy subjects, respectively. The energy of discrete wavelet transform coefficient is derived by the simple equation of energy, energy = ∑_*i*=1_^*n*^(*x*)^2^/*n*. Here, *n* = no.of heart sample. *x* = signal amplitude. We plot the energy for each healthy and unhealthy sample in Figures 23 and 24 and find out the threshold value of 2*e* − 08 to 0.5*e* − 05 for differentiating between them. Threshold values of variance, absolute mean, and energy of DWT for differentiating normal and abnormal signals have been shown in Table 1. It is seen that unhealthy samples' energy is much lower than the energy of healthy samples. A similar result has been found in [32]. So, this energy is being counted as a differentiating factor between healthy and unhealthy samples of the heart sound.

## 5. Conclusion

Body auscultation is now a key and useful human health assessment clinical diagnostic procedure. For automated detection of cardiac diseases, this study introduced heart sound analysis for differentiation of heart sounds collected from normal and abnormal subjects using an IoT device. Features derived from signal amplitude distribution in the time domain and frequency domain analysis reveal that mean frequency is discriminatory enough to distinguish normal and abnormal hearts. The experiment's findings indicate adequate heart sound characteristic differentiation for automated cardiac issue screening employing signal processing from healthy/unhealthy heart sounds. The mean threshold level is found about 0.06-0.09. Above the threshold value is the healthy subject, and below the threshold value is the unhealthy subject. To derive discriminatory features from wavelet heart sound coefficients, the heart sound signal was converted into the wavelet domain.

## 6. Future Work

An advanced IoT-based system can be improved so that the data collected from far areas can easily be transferred to the server to do the analysis. Then, update information about the health condition could be supplied to a person. If we find any abnormality, we can check it earlier before it gets worse. Many transform techniques can be used for further extraction of different features in the biomedical field. Artificial intelligence can be used in this sector for better output and discriminatory features. Machine learning can also be used for the accurate diagnosis of cardiac diseases from heart sounds.

## Figures and Tables

**Figure 1:** Working overview of the proposed system.

**Figure 2:** Complete designed model.

**Figure 3:** (a–e) Successive denoising process using soft thresholding.

**Figure 4:** Amplitude distribution and comparison between healthy and unhealthy heart sound signals.

**Figure 5:** Spectrogram of heart sound recorded from a healthy subject.

**Figure 6:** Spectrogram of heart sounds recorded from an unhealthy subject.

**Figure 7:** Plot of probability distribution of heart sound recorded from a healthy subject.

**Figure 8:** Plot of probability distribution of heart sound recorded from an unhealthy subject.

**Figure 9:** Denoised detailed coefficient using Sym4 level 4 of a healthy subject.

**Figure 10:** Denoised detailed coefficient using Sym4 level 4 of an unhealthy subject. 4 levels of wavelet coefficient before denoising.

**Figure 11:** Detailed coefficient before denoising the signal of a healthy subject.

**Figure 12:** Detailed coefficient before denoising the signal of an unhealthy subject. 4 levels of wavelet coefficient after denoising.

**Figure 13:** Detailed coefficient after denoising the signal of a healthy subject.

**Figure 14:** Detailed coefficient after denoising the signal of an unhealthy subject.

**Figure 15:** Denoised approximation coefficient using Sym4 level 4 of a healthy subject.

**Figure 16:** Denoised approximation coefficient using Sym4 level 4 of an unhealthy subject. 4 levels of wavelet coefficient before denoising.

**Figure 17:** Approximation coefficient before denoising the signal of a healthy subject.

**Figure 18:** Approximation coefficient before denoising the signal of an unhealthy subject. 4 levels of wavelet coefficient after denoising.

**Figure 19:** Approximation coefficient after denoising the signal of a healthy subject.

**Figure 20:** Approximation coefficient after denoising the signal of an unhealthy subject.

**Figure 21:** Mean value (absolute) of healthy and unhealthy subject.

**Figure 22:** Variance comparison of healthy and unhealthy sound.

**Figure 23:** Energy of DWT coefficient of healthy and unhealthy subjects. Unhealthy subjects in detailed view.

**Figure 24:** Detailed view of energy of DWT coefficient of unhealthy subjects.

**Table 1:** Range of threshold for automatic cardiac disorder detection to distinguish between normal and abnormal heart sounds.

Features	Maximum value of abnormal samples for threshold selection	Minimum value of Normal samples for threshold selection	Range for threshold	Feature considered for separation of healthy and unhealthy heart sounds
Absolute mean: signal amplitude	0.07	0.09	0.07-0.09	Yes
Variance	0.01	0.015	0.01-0.015	Yes
Energy of DWT	2*e* − 08	0.5*e* − 05	2*e* − 08–0.5*e* − 05	Yes

## Data Availability

Data can be found in this given repository link https://github.com/amzadjony96/Heart-Sound-Analysis or contact this email amzad.hossain01@northsouth.edu.
